# MiR-19b-3p Attenuates Chondrocytes Injury by Inhibiting MAPK/NF-Κb Axis via Targeting SOCS1

**DOI:** 10.1155/2022/5133754

**Published:** 2022-10-11

**Authors:** Liang Shi, Liang Duan, Dapeng Duan, Yayi Fan, Honghai Xu

**Affiliations:** Department of Orthopedics, Shaanxi Provincial People's Hospital, Xi'an 710068, Shaanxi, China

## Abstract

In this study, miR-19b-3p was downregulated in osteoarthritic cartilage tissues and IL-1*β*-stimulated primary chondrocytes, and miR-19b-3p overexpression reversed the inhibitory effect of IL-1*β* on cell viability, the promotion effects of apoptosis, inflammatory factor secretion and extracellular matrix degradation, whereas the opposite effect was observed with miR-19b-3p inhibitor. Moreover, SOCS1 is a target gene of miR-19b-3p. Furthermore, SOCS1 overexpression enhanced cell injury compared with IL-1*β* alone treatment, whereas knockdown of SOCS1 restored cell damage caused by IL-1*β*. Further studies revealed that miR-19b-3p promoted chondrocyte injury repair by suppressing SOCS1 expression, and we found that was mediated by blocking the MAPK/NF-*κ*B axis. Taken together, our findings may provide a new therapeutic strategy for osteoarthritis.

## 1. Introduction

Osteoarthritis is a progressive degenerative joint disease with a primary predilection for the elderly. The clinicopathological manifestations of osteoarticular cartilage degeneration include apoptosis of chondrocytes as well as disturbances in extracellular matrix (ECM) synthesis, catabolism and metabolism. The relevant epidemiological findings showed that symptomatic knee osteoarthritis was more common in middle-aged and elderly people, with an overall prevalence of 8.1%, and it was significantly higher in women than in men [1]. Concomitant with the accelerating ageing society, there is an increasing trend in the prevalence of osteoarthritis, with the incidence of knee osteoarthritis being as high as more than 50% in the population over the age of 65 years. At present, the main therapeutic measures against osteoarthritis are still to reduce pain and control symptoms, and there is no obvious means to reverse the progression of the disease, so research aimed at osteoarthritis prevention and treatment is becoming more urgent [2].

MicroRNAs (miRNAs), a kind of short chain ribonucleic acid without coding function, can exist in various living bodies. Mature miRNAs suppress the expression levels of corresponding proteins by interfering with the translation process of their target genes, thus achieving sink expression of target genes post transcriptionally [3, 4]. Numerous studies indicating that multiple chronic inflammatory diseases including osteoarthritis may be associated with dysregulation of miRNA expression. MiR-9 functions to regulate MMP-13, and overexpression of miR-9 effectively reduces MMP-13 expression and decreases the level of cartilage matrix degradation [5]. Similarly, knockdown of miR-98 or overexpression of miR-146 in isolated human chondrocytes reduced IL-1*β*-induced TNF-*α* production [6]. MiR-140-5p is an important small nucleic acid molecule involved in maintaining chondrocyte homeostasis, and studies have found that miR-140-5p expression decreases articular cartilage degeneration and aging, and miR-140-5p protect artilage may be achieved by downregulating the corresponding target gene expression, such as ADAMTS5, MMP-13, and IGFBP5 [7].

Recently, emerging evidence has suggested that miR-19b-3p may be involved in the progression of osteoarthritis. Li et al. showed that miR-19b-3p expression was upregulated in osteoarthritic cartilage tissue and IL-1*β* stimulated chondrocytes compared with the control group, and miR-19b-3p mimic inhibited IL-1*β* induced chondrocyte apoptosis and ECM degradation [8]. In addition, a microarray analysis pointed to circulating miR-19b-3p as an independent factor for the risk of knee osteoarthritis, and the combined detection of the remaining miR-122-5p and miR-486-5p may serve as novel biomarkers for the diagnosis of osteoarthritis [9]. Independently, another study found that miR-19b-3p mimic significantly increased chondrocyte viability and inhibited apoptosis, it also increased the expression of type II collagen, aggrecan and glycosaminoglycan, and decreased the expression of MMP-1 and MMP-13 caused by IL-1*β*, suggesting that miR-19b-3p is able to attenuate osteoarthritis injury [10].

Therefore, we used miR-19b-3p as an entry point to deeply explore the potential mechanism of miR-19b-3p to inhibit chondrocyte matrix degradation and delay the progression of osteoarthritis, with a view to improving new references for osteoarthritis treatment.

## 2. Materials and Methods

### 2.1. Cell Culture

Articular cartilage tissue was collected and fully digested in DMEM with streptomycin and collagenase, and then the digested material was filtered to obtain the culture medium. Next, the medium was centrifuged (1000 r/min; 5 min) and the supernatant discarded, and DMEM (containing FBS, penicillin, and streptomycin) was added again. Cells were cultured in culture bottle (2 × 10^5^) and rested in an incubator with 5% CO_2_ at 37°C. The protocol of this study was approved by the ethics committee of Shaanxi Provincial People's Hospital, and written informed consent was obtained from each participant. The miR-19b-3p mimic, miR-19b-3p inhibitor and their negative control were performed from RiboBio Co., Ltd. The pcDNA-SOCS1 and vector were purchased from RiboBio Co., Ltd. The si-SOCS1 and scramble were purchased from Santa Cruz Biotechnology. SiRNAs targeting SOCS1 (sense 5′ UCG CCC UUA GCG UGA AGA U 3′; antisense 5′ AUC UUC ACG CUA AGG GCG A 3′), and scramble sequence siRNA (sense 5′ UCG AUU CUG CGA AGC CGA U 3′; antisense 5′ AUC GGC UUC GCA GAA UCG A 3′).

### 2.2. RT-qPCR

Cell Total RNA was isolated by the TRIzol. Single-stranded cDNA was synthesized with the PrimeScript Reagent Kit. Real-time qPCR was conducted by using a SYBR Premix Ex TaqTM Kit. Sangon Biotech designed and costained the primers in the study. MiR-19b-3p forward, 5′-CAC TGT TCT ATG GTT AG-3′, reverse, 5′-CAC TAC CAC AGT CAG TT -3′'; SOCS1 forward, 5′- CTT CCT CCT CTT CCT CCT C-3′, reverse, 5′- GCC ATC TTC ACG CTA AGG-3. The relative expression levels were normalized by using the 2^−ΔΔCt^ method.

### 2.3. Western Blotting

Cell protein were extracted by RIPA lysis buffer. Next, proteins were transferred to PVDF membranes and blocked for 2 h at room temperature and incubated at primary antibodies for 12 h. GAPDH (1 : 3000), SOCS1 (1 : 1000), cleaved caspase3 (1 : 500), MAPK (1 : 2000), MAPK (phospho Y322, 1 : 500), NF-*κ*B (1 : 1500) and NF-*κ*B (phospho S337, 1 : 1000). Then, the membranes were incubated with secondary antibody (1 : 2500, ab6721) for 1 h. Next, an exposure liquid is added and a visualized protein band is acquired in the instrument. The bands were visualized by using an ECL Plus Chemiluminescence Reagent Kit (Pierce, Rockford, IL, USA) and were photographed by a chemiluminescence imaging system. Image J software was used to quantify the band densities.

### 2.4. CCK-8 Assay

The cells were digested with 0.25% trypsin, and then the cell suspension (3 × 10^4^/mL) was prepared again with DMEM, and then inoculated into 96-well plates (100 *μ*L), and incubated for 4 h (37°C; 5% CO_2_). The absorbance was measured by a microplate reader (450 nm).

### 2.5. ELISA

The secretion levels of IL-6, TNF-*α*, COX-2, MMP13, collagen II and ADAMTS5 were detected by ELISA kit (Solarbio, China).

### 2.6. Flow Cytometry

The cell suspension (100 *μ*L, 1 × 10^5^ cells/mL) was prepared with PBS and transferred to the culture tube, and then cultured with annexin V-FITC and propidium iodide in a dark environment for 20 min. Finally, apoptotic cells were determined by flow cytometry.

### 2.7. Luciferase Reporter Gene Assay

First, SOCS1 wild- and mutant-type sequences were fused in a PGL3 luciferase reporter vector. Next, miR-19b-3p mimic and negative control were transfected into HEK293 cells together with luciferase reporter vectors, and after 48 h of culture, luciferase activity was measured by a microplate reader (MA, USA).

### 2.8. Statistical Analysis

The SPSS software was used to analysed all dates (ver. 21.0). The quantitative data derived from three independent experiments were expressed as mean ± SD. *P* < 0.05 means statistically significant.

## 3. Results

### 3.1. MiR-19 b-3p Alleviates the Damage of IL-1*β*-Treated Chondrocytes

The miR-19b-3p expression was downregulated in osteoarthritic cartilage tissues (Figure 1(a)). Next, the transfection efficiency of miR-19b-3p is shown in Figure 1(b). Then, the cell viability was inhibited (Figure 1(c)) and apoptosis (Figure 1(d)), inflammatory factor secretion (Figure 1(e)), and extracellular matrix degradation was promoted after IL-1*β* treatment (Figure 1(f)), as indicated by increased secretion of MMP-13 and ADAMTS5 and decreased secretion of type 2 collagen, whereas overexpression of miR-19b-3p aggravated chondrocyte injury caused by IL-1*β*, and transfection of miR-19b-3p inhibitor had the opposite effect.

### 3.2. SOCS1 was a Direct Target of miR-19b-3p

Figure 2(a) showed the SOCS1 wild- and mutant-type sequences, respectively (https://starbase.sysu.edu.cn/). Next, miR-19b-3p mimic decreased the luciferase activity of SOCS1 wild-type reporter, instead of SOCS1 mutant reporter (Figure 2(b)). Moreover, miR-19b-3p mimic decreased SOCS1 mRNA and protein expression), and miR-19b-3p inhibitor increased SOCS1 mRNA (Figure 2(c)) and protein (Figure 2(d)) expression.

### 3.3. SOCS1 Aggravates the Damage of IL-1*β*-Treated Chondrocytes

The pcDNA-SOCS1 and si-SOCS1 were transfected into IL-1*β*-treated chondrocytes. IL-1*β* promoted SOCS1 protein expression, and SOCS1 overexpression enhanced the effect of IL-1*β*, whereas knockdown of SOCS1 expression had the opposite effect (Figure 3(a) and 3(b)). Moreover, compared with IL-1*β* treated, the pcDNA-SOCS1 inhibited cell viability (Figure 3(c)), promoted the expression of apoptosis related protein cleaved caspase3 (Figure 3(a) and 3(d)), inflammatory factors secretion (Figure 3(e)) and extracellular matrix degradation (Figure 3(f)), and si-SOCS1 alleviated cell damage caused by IL-1*β*.

### 3.4. MiR-19 b-3p Alleviates IL-1*β*-Induced Chondrocyte Injury by Inhibiting SOCS1

We observed that overexpression of miR-19b-3p inhibited SOCS1 expression compared with IL-1*β* treatment, whereas transfection of pcDNA-SOCS1 inhibited SOCS1 expression (Figure 4(a)). Furthermore, miR-19b-3p mimic enhanced cell viability (Figure 4(b)) and decreased cell injury (Figure 4(c), 4(d) and 4(e)) compared with IL-1*β* alone treatment, and pcDNA-SOCS1 reversed the protective effect.

### 3.5. MiR-19 b-3p Attenuates IL-1*β*-Induced Chondrocyte Injury via MAPK/NF-Κb Signaling Pathway

We found that IL-1*β* increased p38 MAPK phosphorylation levels, promoted NF-*κ*B p65 protein expression, and miR-19b-3p overexpression reversed this effect, and C16-PAF (MAPK pathway) reversed the effect of miR-19b-3p (Figure 5(a) and 5(b)). Furthermore, miR-19b-3p mimic decreased apoptotic protein cleaved caspase3 expression (Figure 5(a) and 5(c)), inflammatory factor secretion (Figure 5(d)), and extracellular matrix degradation (Figure 5(e)), but this protective effect on chondrocytes was abolished by MAPK activator.

## 4. Discussion

Suppressors of cytokine signaling (SOCS) are a recently identified class of protein signaling molecules that function prominently in the immune system by inhibiting cytokine signaling through negative feedback loops. SOCS1 plays important roles in various physiopathological processes, such as cell differentiation, regulation of inflammation, participation in tumor immunity, and regulation of metabolism. He et al. showed that SOCS1 knockdown increased osteoarthritic chondrocytes viability [11]. In rheumatoid arthritis progression, silencing SOCS1 has been reported to promote cell proliferation and invasion, upregulate IL-1*β* and MMP expression, and activate the ERK pathway to alleviate synovial tissue damage [12].

Osteoarthritis is characterized by an imbalance in ECM synthesis and degradation, resulting in joint pain and progressive dysfunction. Numerous factors are involved in cartilage destruction in osteoarthritis, mainly cytokines or chemokines including TNF and IL, inflammatory mediators including PGE2 and NO, MMP-13 and components of degraded matrix including ADAMTS [13, 14]. The MMPs family consists of 20 different enzymes whose expression levels are significantly higher in osteoarthritis than in normal cartilage, and the expression of MMP-13 in normal cartilage is only one fourth of its expression in osteoarthritic chondrocytes. MMP-13, a member of the extracellular matrix degrading endopeptidase family, is a key MMP collagen hydrolase because it degrades collagen and a wide range of matrix molecules [15, 16].

As early as 1994, the p38 MAPK axis was found to be involved in the physiological response of yeast to stress stimuli in fungal studies, and it is also involved in the inflammatory response and stress stimuli in mammals. A variety of studies have now shown MAPKs signaling activation in osteoarthritic cartilage tissue, manifested by increased levels of p38 MAPK, ERK as well as JNK phosphorylation [17–20]. In addition, the NF-*κ*B signaling pathway exists widely in various cells, mainly in the inactive p65 subunit form, and phosphorylation occurs when p65 is activated, whereas p65 transduces into the nucleus after dissociation from the phosphoproteasome, further activating the inflammatory response and secreting a series of proinflammatory cytokines [21]. In a word, miR-19b-3p promotes viability, inhibits apoptosis, and reduces inflammatory factor secretion and extracellular matrix degradation of injured chondrocytes by targeting and inhibiting SOCS1 expression, and this is mediated by blocking the MAPK/NF-*κ*B axis.

## Figures and Tables

**Figure 1:** Effect of miR-19b-3p on chondrocytes (a) The miR-19b-3p expression in tissues (b) MiR-19 b-3p expression (c) Cell viability (d) Cell apoptosis (e) Levels of inflammatory factor secretion (f) The secretion levels of MMP-13, Collagen II and ADAMTS5. ^*∗*^*P* < 0.01.

**Figure 2:** SOCS1 is a direct target of miR-19b-3p. (a). SOCS1 sequences (wild- and mutant-type). (b). Relative luciferase activity (wild- and mutant-type of SOCS1). C&D. SOCS1 mRNA and protein expression. ^*∗*^*P* < 0.01.

**Figure 3:** Effect of SOCS1 on chondrocytes. a&b. SOCS1 protein expression. (c) Cell viability. a&d. Cleaved caspase3 protein expression. (e) Levels of inflammatory factor secretion. (f) MMP-13, Collagen II and ADAMTS5 secretion levels. ^*∗*^*P* < 0.01.

**Figure 4:** MiR-19 b-3p affects chondrocytes via SOCS1. (a) SOCS1 protein expression. (b) Cell viability. (c) Cell apoptosis. (d) Levels of inflammatory factor secretion. (e) MMP-13 and Collagen II secretion levels. ^*∗*^*P* < 0.01.

**Figure 5:** MiR-19 b-3p affects chondrocytes through the MAPK/NF-*κ*B axis. a&b. The phosphorylation of p38 MAPK and NF-*κ*B p65 protein. a&c. Cleaved caspase3 protein expression. (d) Inflammatory factor secretion levels. (e) The secretion levels of Collagen II and ADAMTS5. ^*∗*^*P* < 0.01.

## Data Availability

The labeled dataset used to support the findings of this study are available from the corresponding author upon request.
